This article has been retracted.

# TLE3 represses colorectal cancer proliferation by inhibiting MAPK and AKT signaling pathways

**DOI:** 10.1186/s13046-016-0426-8

**Published:** 2016-09-27

**Authors:** Run-Wei Yang, Ying-Yue Zeng, Wen-Ting Wei, Yan-Mei Cui, Hui-Ying Sun, Yue-Long Cai, Xin-Xin Nian, Yun-Teng Hu, Yu-Ping Quan, Sheng-Lu Jiang, Meng Wang, Ya-Li Zhao, Jun-Feng Qiu, Ming-Xuan Li, Jia-Huan Zhang, Mei-Rong He, Li Liang, Yan-Qing Ding, Wen-Ting Liao

**Affiliations:** 1 Department of Pathology, Nanfang Hospital, Southern Medical University, Guangzhou, 510515 Guangdong China; 2 Department of Pathology, School of Basic Medical Sciences, Southern Medical University, Guangzhou, Guangdong China; 3 Guangdong Provincial Key Laboratory of Molecular Tumor Pathology, Guangzhou, Guangdong China; 4 Guangdong Provincial Key Laboratory of Gastroenterology, Department of Gastroenterology, Nanfang Hospital, Southern Medical University, Guangzhou, Guangdong China; 5 Department of Pathology, Nanfang Hospital and School of Basic Medical Sciences, Southern Medical University, Guangzhou, 510515 Guangdong China

**Keywords:** TLE3, Proliferation, Prognosis, Colorectal cancer, p21Cip1/WAF1, p27Kip1

## Abstract

**Background:**

Transducin-like enhancer of Split3 (TLE3) serves as a transcriptional corepressor during cell differentiation and shows multiple roles in different kinds of cancers. Recently, TLE3 together with many other genes involved in Wnt/β-catenin pathway were detected hyper-methylated in colorectal cancer (CRC). However, the potential role and the underlying mechanism of TLE3 in CRC progression remain scarce.

**Methods:**

Gene expression profiles were analyzed in The Cancer Genome Atlas (TCGA) microarray dataset of 41 normal colorectal intestine tissues and 465 CRC tissues. Western blot and Real-time Quantitative PCR (RT-qPCR) were respectively performed to detect protein and mRNA expression in 8 pairs of CRC tissue and matched adjacent normal mucosa. Immunohistochemistry (IHC) was conducted to evaluate TLE3 protein expression in 105 paraffin-embedded, archived human CRC tissues from patients, whose survival data were analyzed with Kaplan-Meier method. In vitro experiments including MTT assay, colony formation assay, and soft agar formation assay were used to investigate the effects of TLE3 on CRC cell growth and proliferation. Additionally, subcutaneous tumorigenesis assay was performed in nude mice to confirm the effects of TLE3 in vivo. Furthermore, gene set enrichment analysis (GSEA) was run to explore potential mechanism of TLE3 in CRC, and then we measured the distribution of CRC cell cycle phases and apoptosis by flow cytometry, as well as the impacts of TLE3 on MAPK and AKT signaling pathways by Western blot and RT-qPCR.

**Results:**

TLE3 was significantly down-regulated in 465 CRC tissues compared with 41 normal tissues. Both protein and mRNA expressions of TLE3 were down-regulated in CRC compared with matched adjacent normal mucosa. Lower expression of TLE3 was significantly associated with poorer survival of patients with CRC. Besides, knock down of TLE3 promoted CRC cell growth and proliferation, while overexpression of TLE3 showed suppressive effects. Furthermore, overexpression of TLE3 caused G1-S phase transition arrest, inhibition of MAPK and AKT pathways, and up-regulation of p21Cip1/WAF1 and p27Kip1.

**Conclusion:**

This study indicated that TLE3 repressed CRC proliferation partly through inhibition of MAPK and AKT signaling pathways, suggesting the possibility of TLE3 as a biomarker for CRC prognosis.

**Electronic supplementary material:**

The online version of this article (doi:10.1186/s13046-016-0426-8) contains supplementary material, which is available to authorized users.

## Background

Colorectal cancer (CRC) is one of the most commonly studied malignancies because of high morbidity and mortality [1]. CRC carcinogenesis is a multistep progress involving progressive genetic mutations, epigenetic adaptation, and immunology aberrances [2–4], which lead to the complexity of clinical treatment. Although continuous progresses were obtained in diagnostic and therapeutic methods, the prognosis and outcome of CRC patients are far away from satisfaction [5]. Recent studies intensively focus on personalized therapy that requires efficient biomarkers capable of assisting early diagnosis and treatment [6, 7]. However, current biomarkers of CRC are unmet [8, 9].

Groucho (Gro)/TLE proteins belong to a large family of transcriptional corepressor that are extensively expressed in most metazoans. They show high conservation in structure and function of C-terminal tryptophan–aspartate (WD)-repeat domain and N-terminal glutamine-rich (Q) domain [10]. After direct interaction with DNA-bound transcriptional factors through WD-repeat domain, the Gro/TLE proteins form into polymer via Q domain with each other along the chromosome, and then recruit histone deacetylases to establish a transcriptionally silenced chromatin structure [10–12]. This complex exerts long-range repression on a variety of transcriptional factors including the members of Hes, Runx, Lcf/Lef, Pax, Six, and c-Myc families [11, 13]. In this way, the Groucho/TLE proteins participate in receptor tyrosine kinase (RTK)/Ras/Ral, mitogen-activated protein kinase (MAPK), Notch, Wnt, and Hedgehog signaling pathways during processes of embryonic development, morphogenesis and cell metabolism, as well as neoplastic conditions [10, 14–18].

Transducin-like enhancer of Split 3 (TLE3) is one of the full-length members of human TLE family [19]. Besides dynamic functions in differentiation and cell metabolism [15, 20–22], TLE3 emerges attractive property in tumorigenesis. It was initially found elevated in cervical and colonic neoplasms [23, 24]. However, methylation status analyses of colorectal tumors showed aberrant methylation in the CpG island of TLE3 when compared with adjacent normal mucosa [25]. Additionally, altered expression of TLE2 and TLE3 were associated with high-grade meningioma [26], and the alternatively spliced isoforms of TLE3 were detected upregulated in prostate tumor [27, 28]. TLE3 was indifferent in leukemia, although other TLE proteins were observed coordinating with FOXG1 to promote B-lineage leukemia of positive E2A-HLF oncoprotein [29]. Interestingly, several studies proposed TLE3 as a potential marker of taxane responsiveness in the treatment of ovarian carcinoma and breast cancer [30, 31], but the most recent NCIC CTG MA.21 clinical trial repudiated TLE3 to be a valuable marker for taxane sensitivity in breast cancer treatment [32]. In short, these findings revealed the erratic role of TLE3 in human cancers. Further investigation of TLE3’s pathological characteristics and clinical application in CRC will be of great significance.

Here, we sought to explore the expression pattern and potential role of TLE3 in the progression of CRC. Our study showed that TLE3 expression was significantly down-regulated in CRC tissue than matched adjacent normal mucosa. Lower expression level of TLE3 was associated with poorer outcome of CRC patients. Furthermore, TLE3 could arrested cell cycle progression and suppressed cell proliferation as well as tumor growth in CRC partially through inhibition of MAPK and AKT pathways.

## Methods

### Patients and specimens

A total of 105 pathological specimens were obtained from colon cancer patients between 2009 and 2014 at the Department of Pathology, Nanfang Hospital Southern Medical University. Medical records of these patients provided information of gender, age, and following essential factors: tumor pathological characteristics, pathologic stage, T stage, Dukes stage, metastases of lymph node, and distant metastasis. The 8 pairs of fresh biopsies collected from CRC and their matched noncancerous mucosa tissue were obtained from the operation room of Nanfang Hospital. The fresh biopsies were stored in liquid nitrogen before usage. Approval was obtained from the Southern Medical University Institutional Board (Guangzhou, China) for the use of clinical materials for research purposes. All samples were collected and analyzed with the prior written, informed consent of the patients.

### Cell cultures

The human CRC cell lines SW480, Ls174t, HCT15 and SW620 were purchased from American Type Culture Collection. SW620 were cultured in DMEM medium (Gibco) supplemented with 10 % fetal bovine serum (FBS) (PAA Laboratories, Pasching, Austria). Ls174t, HCT15 and SW480 were cultured in RPMI 1640 medium (Gibco) with 10 % FBS. Dissolved by DMSO, ERK inhibitor GDC0994 (50 μM) and AKT inhibitor PF04691502 (10 μM) (Selleck Chemicals, USA) were used to inhibit the activation of MAPK and AKT pathways, respectively. Cells were cultured at 37 °C with 5 % CO_2_.

### Plasmids

The full-length TLE3 was amplified by PCR and cloned into pBabe (Addgene, Inc., Cambridge, MA, USA). The human short hairpin RNA (shRNA) sequences specifically targeting TLE3 (TLE3 shRNA#1: 5′-CCACACGTTTGCAACCCAA-3′; TLE3 shRNA#2: 5-CCTCCTGGTATCTGAACCA-3′) were cloned into pSuper-retroneo (Oligo-Engine, Seattle, WA, USA).

### RNA isolation, reverse transcription (RT) and Real-time Quantitative PCR (RT-qPCR)

Total RNA from cultured cells and CRC tissues was isolated using the mirVana miRNA Isolation Kit (Ambion) according to the manufacturer’s instruction. The cDNA was then synthesized from total RNA using the Taqman miRNA reverse transcription kit (Applied Biosystems, Foster City, CA, USA). RT-qPCR was performed with the Applied Biosystems 7500 Sequence Detection system, using iQ™ SYBR Green Supermix (BioRad Laboratories, Hercules, CA, USA). The data were normalized to the geometric mean of housekeeping gene GAPDH values and calculated as 2^−ΔΔCT^ method. Sequences of the primers for RT-qPCR are summarized in Additional file 1: Table S1.

### Western blot

We carried out western blot as previously described [33], using anti-TLE3 (Abcam, Cambridge, MA, USA), anti-FOXO3, anti-Akt, anti-GSK-3β, anti-ERK, anti-p21, anti-p27, anti-p-FOXO3, anti-p-Akt, anti-p-GSK-3β and anti-p-ERK (Bioworld Technology, St. Louis Park, MN, USA) to detect the corresponding proteins. Anti-α-Tubulin monoclonal antibody (Sigma, St. Louis, MO, USA) served as a loading control.

### Immunohistochemistry

Immunohistochemistry (IHC) staining and scoring were performed as previously described [33]. Ki-67 detected by anti-Ki-67 (Abcam, Cambridge, MA, USA) represented the proliferation index.

### MTT assay

Cells were incubated for 24 h at 37 °C after the cells were trypsinized and plated on 96-well plates (1 × 10^3^). Then 20 μl of 5 g/L MTT (3-(4, 5-dimethylthiazol-z-yl)-2, 5-diphenyltetrazolium bromide, Sigma, St. Louis, MO, USA) was added and mixed into each well and incubated at 37 °C. After 4 h, the MTT-medium mixture was removed and 150 μl dimethyl sulphoxide (DMSO, Sigma, St. Louis, MO, USA) were added into the wells. The absorbance value was measured at 490 nm with a Microplate Autoreader (Bio-Rad, Hercules, CA, USA). Three dependent experiment was repeated. Data were presented as the mean ± SD.

### Colony formation assay

Cells (200 cells/well) were trypsinized and plated on 6-well plates, and then cultured in medium with 10 % FBS for 2 weeks. The colonies were fixed with 4 % paraformaldehyde for 5 min and stained with 1 % crystal violet for 30 s. Colonies of more than 50 cells were counted. The experiment was repeated for 3 times independently. Data were presented as the mean ± SD.

### Soft agar assay

60 mm plates were covered with a layer of 0.66 % agar in medium supplemented with 20 % FBS. Cells (1 × 10^4^) were seeded on the top of agar layer and cultured in RPMI 1640 supplemented with 10 % FBS with 0.3 % agarose. The cells were incubated with 5 % CO_2_ at 37 °C. After 2 to 3 weeks, the number of cell colony were counted under microscope and cell colonies were photographed in 100 × view. Colonies of more than 50 cells were counted. The experiment was repeated for 3 times independently, each cell line respectively. Data were presented as the mean ± SD.

### Cell cycle analysis

Cell cycle distribution was examined by measuring the cellular DNA content using flow cytometry. Cells at 80–90 % confluence were incubated for 36 h in the RPMI-1640 medium containing 0.5 % FBS, then released through culturing back in RPMI-1640 medium with 10 % FBS for 12 h. 1 × 10^6^ cells were collected and fixed with 70 % cold ethanol. After treated with RNase A (10 μg/mL) for 30 min at 37 °C, the cells were resuspended in 0.5 mL propidium iodide (PI) solution (50 μg/mL in 0.1 % sodium citrate with 0.1 % NP-40). Cell cycle distribution was analyzed by FACScan cytometry (Becton-Dickinson, San Jose, CA, USA).

### Tumorigenesis assay

Cells were trypsinized and then suspended with serum-free medium. 200 μl cell suspension (2 × 10^6^ cells) was subcutaneously injected into 4-week-old Balb/Cathymic nude mice (nu/nu) obtained from the Animal Center of Southern Medical University, Guangzhou, Guangdong Province, China. All the animals were housed and maintained under specific pathogen-free conditions, and all experiments were approved by the Use Committee for Animal Care and performed in accordance with institutional guidelines. Tumor volumes were measured on the indicated days. Tumor size was measured by a slide caliper and tumor volume was determined by the formula 0.44 × A × B^2^ (A indicates tumor base diameter one direction and B the corresponding perpendicular value). The tumors were fixed and 4 μm sections were cut and stained with haematoxylin and eosin according to standard protocols. Sections were further under IHC staining using antibody against Ki-67.

### Statistical analysis

All statistical analyses were carried out using SPSS version 19.0 for Windows (IBM, Armonk, NY, USA). The two-tailed Student’s *t*-test was used to compare the intergroup. Survival data were analyzed with Kaplan-Meier method and were compared using the log-rank test. *p* < 0.05 was considered statistically significant.

## Results

### Down-regulation of TLE3 was associated with advanced progression and poor survival of human CRC

In order to identify deregulated genes involved in the progression of CRC, gene expression profiles were analyzed in The Cancer Genome Atlas (TCGA) microarray datasets. The analyses showed that TLE3 was significantly down-regulated in 465 CRC tissues compared to 41 normal tissues (Fig. 1a and b). Consistent with this finding, Western blot and real-time PCR analyses showed that TLE3 expression was significantly down-regulated in eight CRC tissues compared with adjacent normal intestine epithelial tissues (Fig. 1c and d). Furthermore, TLE3 protein expression was detected by immunohistochemistry (IHC) in 105 paraffin-embedded, archived human CRC tissues. TLE3 protein expression was quite abundant in adenoma as well as normal tissue, whereas it was markedly decreased in adenocarcinoma (Fig. 1e). Kaplan-Meier survival analysis showed that CRC patients with lower level of TLE3 protein expression had a poorer prognosis (Fig. 1f). These results suggest that TLE3 down-regulation is significantly associated with advanced progression of human CRC.

**Fig. 1:** Evaluation of TLE3 expression in CRC cell lines and primary human CRC. **a** Analyses of TLE3 expression in normal colorectal intestines (*n* = 41) and colorectal tumors (*n* = 465) in The Cancer Genome Atlas (TCGA) microarray dataset. **b** Analyses of TLE3 expression in 41 pairs of tissues of normal colorectal intestines and colorectal tumors in TCGA microarray dataset. **c** Expression of TLE3 protein in 8 primary human CRC tissue (T) and the adjacent normal tissue (N) paired from the same patient by Western blot. **d** Real-time PCR was used to quantify average N/T ratios of TLE3 mRNA expression. **e** Representative images of TLE3 protein expression in normal colorectal epithelia, adenoma and adenocarcinoma by IHC. TLE3 was positively detected in both adenoma and their adjacent normal tissue (*middle and left*), whereas there was little detection in adenocarcinoma (*right*). **f** Influence of TLE3 expression on overall survival by Kaplan-Meier analysis in 105 patients with CRC. *p* < 0.05 The expression levels of protein or mRNA were normalized with α-Tubulin or GAPDH, respectively. Error bars represent mean ± SD calculated from 3 independent experiments

### Overexpression of TLE3 repressed the proliferation and tumorigenesis of human CRC cells

To investigate the potential role of TLE3 in the progression of human CRC, stable CRC cell lines SW480 and Ls174t of TLE3 overexpression were established (Fig. 2a). In comparison with control cells, the proliferation of SW480 and Ls174t cells was inhibited by TLE3 overexpression as determined by MTT and colony formation assays (Fig. 2b and c). Anchorage-independent growth activity was examined using soft agar formation assays, whose results showed that TLE3 overexpression also repressed the proliferation of SW480 and Ls174t cells in soft agar, as both the number and size of colonies were decreased in comparison with control cells (Fig. 2d). To confirm this effect in vivo, tumorigenesis assays by subcutaneous injection were performed in nude mice. The TLE3 overexpression group exhibited remarkably slower tumor growth and smaller tumor volume in comparison with the control group (Fig. 2e, *n* = 6). In addition to the difference of tumor volume, much lower Ki-67 index was found in tumors formed by TLE3 overexpression group than that in the control group, as detected by IHC analysis of Ki-67 (Fig. 2f).

**Fig. 2:** Overexpression of TLE3 repressed the proliferation and tumorigenesis of human CRC cells. **a** Overexpression of TLE3 in SW480 and Ls174t cells. α-Tubulin was used as a loading control. **b** Overexpression of TLE3 repressed cell proliferation of SW480 and Ls174t cells by MTT assays. **c** Overexpression of TLE3 repressed cell proliferation of SW480 and Ls174t cells by colony formation assays. **d** Overexpression of TLE3 repressed anchorage-independent growth ability of SW480 and Ls174t cells as determined by soft agar assays. Colonies containing more than 50 cells were scored. **e** Tumorigenesis assay by subcutaneous injection of SW480/vector or SW480/TLE3 cells in nude mice (*n* = 6/group). Tumor volumes were measured on the indicated days. Data points are the mean tumor volumes ± SD. *p* < 0.05. **f** The sections of tumor were under H&E staining or subjected to IHC staining using an antibody against Ki-67. Error bars represent the mean ± SD of 3 independent experiments. * *p* < 0.05

### Knock-down of TLE3 promoted the proliferation and tumorigenesis of human CRC cells

To further confirm the role of TLE3 in human CRC cells proliferation, endogenous expression of TLE3 in HCT15 and SW620 was knocked down by specific shRNAs (Fig. 3a). MTT and colony formation assays indicated that knock-down of TLE3 expression obviously promoted the cell growth of HCT15 and SW620 cells in comparison with control cells (Fig. 3b and c). Besides, the number and size of colonies in soft agar assays were significantly increased in TLE3-silenced HCT15 and SW620 cells in comparison with control cells (Fig. 3d). Furthermore, knockdown of endogenous TLE3 expression in SW620 cells led to noteworthy promotion of tumor growth and volume in the tumorigenesis assays by subcutaneous injection in nude mice, confirming the suppressive effect of TLE3 on CRC proliferation in vivo (Fig. 3e; *n* = 6). In contrast to tumors of TLE3 overexpression, Ki-67 index was found much higher in tumors of TLE3 knock-down in comparison with control cell-based tumor (Fig. 3f).

**Fig. 3:** Knock-down of TLE3 promoted the proliferation and tumorigenesis of human CRC cells. **a** RNAi-silencing of TLE3 in shRNA-transduced stable HCT15 and SW620 cells. α-Tubulin was used as a loading control. **b** Knock-down of TLE3 promoted cell proliferation of HCT15 and SW620 cells by MTT assays. **c** Knock-down of TLE3 promoted cell proliferation of HCT15 and SW620 cells by colony formation assays. **d** Knock-down of TLE3 promoted anchorage independent growth ability of HCT15 and SW620 cells as determined by soft agar assays. Colonies containing more than 50 cells were scored. **e** Tumorigenesis assay by subcutaneous injection of SW620/Scr and SW620/sh-1 cells in nude mice (*n* = 6/group). Tumor volumes were measured on the indicated days. Data points are the mean tumor volumes ± SD. **f** The sections of tumor were under H&E staining or subjected to IHC staining using an antibody against Ki-67. Error bars represent the mean ± SD of 3 independent experiments. * *p* < 0.05

### TLE3 caused cell cycle G1-S phase transition arrest in human CRC cell

To explore the possible mechanism by which TLE3 regulates the proliferation of human CRC cells, we analyzed TLE3 RNA expression levels based on TCGA COAD RNA Seq dataset and cycling gene signatures from the online Gene Set Database of the gene set enrichment analysis (GSEA) [34]. We observed that TLE3 expression was negatively correlated with genes related to cell cycle and G1-S transition (Additional file 2: Figure S1a and b). Furthermore, flow cytometry was performed to measure the distribution of cell cycle phases. Compared with control cells, the percentage of G1-phase cells increased and S-phase decreased significantly in the SW480 cells with TLE3 overexpressing (27.14 vs 41.55 %, *p* < 0.05, and 49.47 vs 34.02 %, *p* < 0.05, respectively) (Fig. 4a and Additional file 3: Figure S2a). Another cell line Ls174t of TLE3 overexpression showed the same results (29.38 vs 51.22 %, *p* < 0.05 and 52.67 vs 41.38 %, *p* < 0.05, respectively) (Fig. 4a and Additional file 3: Figure S2a). On the contrary, decrease in the percentage of G1-phase cells and increase in the percentage of S-phase were observed after endogenous TLE3 in HCT15 and SW620 cells was knocked down. The percentage of S-phase cells in HCT15 and SW620 cells of TLE3 knock-down were significantly more than that in HCT15 and SW620 cells of control group (40.35 vs 50.88 %, *p* < 0.05 and 29.49 vs 39.88 %, *p* < 0.05, respectively) (Fig. 4b and Additional file 3: Figure S2b). Moreover, TLE3 overexpressing significantly increased the percentage of apoptotic cells in SW480 and Ls174t cells, whereas knockdown of TLE3 in SW620 and HCT15 cells decreased the number of apoptotic cells (Fig. 4c and d, Additional file 3: Figure S2c and d). Taken together, these results demonstrate that TLE3 inhibits cell cycle progression and promotes cell death in CRC cells.

**Fig. 4:** TLE3 inhibited cell cycle progression of human CRC cell. **a, b** Representative figures depicting cell cycle profiles of indicated cells. Cells were stained with PI and analyzed by flow cytometry. **c, d** Flow cytometry of annexin V and PI-labelled CRC cells indicating apoptosis

### TLE3 suppressed CRC partly through inhibition of MAPK and AKT signaling pathways

The GSEA analysis based on TCGA COAD RNA expression dataset also revealed that TLE3 level was negatively correlated with AKT activity (Additional file 4: Figure S3), indicating that TLE3 might inhibit the activation of AKT signaling pathway. Moreover, Western blot showed that the levels of phosphorylated FOXO3, GSK, ERK and AKT were decreased in SW480 and Ls174t cells with TLE3 overexpressing, whereas increased in HCT15 and SW620 cells with TLE3 knocking down in comparison with control cells (Fig. 5a). Since TLE3 significantly inhibited the G1-S phase transition as shown above, we then detected the cyclin-dependent kinases inhibitor proteins p21Cip1/WAF1 (p21) and p27Kip1 (p27) that are responsible for this transition [35, 36]. Results showed that p21 and p27 were upregulated in SW480 and Ls174t cells with TLE3 overexpressing (Fig. 5a), whereas they were down-regulated in HCT15 and SW620 cells with TLE3 knocking down (Fig. 5a). Additionally, transcriptional levels of p21 and p27 were also regulated by TLE3 (Additional file 5: Figure S4 a, b, c and d).

**Fig. 5:** TLE3 regulated p21 and p27 through the MAPK and AKT signaling pathways in CRC cells. **a** Western blot analyses of the expression of p-FOXO3a, total FOXO3a, phosphorylated GSK, total GSK, phosphorylated ERK, total ERK, phosphorylated AKT, total AKT, p21Cip1/WAF1 and p27Kip1 proteins in indicated human CRC cell lines. **b** SW620 cells with TLE3 knocking down were treated with the AKT inhibitor PF04691502 (10 μM), the ERK inhibitor GDC0994 (50 μM) or DMSO for 24 h, then harvested to examine the expression levels of the indicated proteins by western blot. **c, d** and **e** Proliferation ability of SW620 cells with TLE3 knocking down was determined by MTT assay (**c**), colony formation assay (**d**) and soft agar assay (**e**) after treatment with GDC0994, PF04691502 or DMSO. Error bars represent mean ± SD from 3 independent experiments. * *p* < 0.05

To investigate whether the alterations of p21 and p27 were caused by activation of the MAPK or AKT pathways, SW620 cells with TLE3 knocking down were treated with an ERK inhibitor (GDC0994)[37] or AKT inhibitor (PF04691502)[38]. Figure 5b showed that the expression levels of phosphorylated ERK and AKT were significantly reduced by GDC0994 and PF04691502 in SW620 cells, respectively. Notably, the expression of p21 and p27 were rescued by treatment with the ERK or AKT inhibitors compared to control cells treated with DMSO (Fig. 5b).

To further confirm that TLE3 represses proliferation by inhibiting the MAPK and AKT pathways, the growth ability of SW620 cells with TLE3 knocking down after treatment with GDC0994 or PF04691502 were examined. MTT assay, colony formation assay and soft agar assay showed that the growth of SW620 cells were significantly compromised by treatment with the ERK or AKT inhibitors compared to control cells treated with DMSO (Fig. 5c, d and e).

Collectively, these results indicate that TLE3 represses the proliferation of CRC cells partly through inhibition of MAPK and AKT signaling pathways and activation of p21 and p27.

## Discussion

Although TLE3 gene was detected hyper-methylated in CRC [25], our study firstly reported the down-regulation of TLE3 on both protein and mRNA levels. Results revealed that low expression of TLE3 in CRC was significantly correlated with advanced progression and poor survival of patients. In addition, TLE3 expression was observed negatively associated with CRC growth both in vitro and in vivo. However, whether TLE3 could be used as a valuable biomarker for CRC prognosis needs further investigation.

The TLE family show structural redundancy [19] but play multiple roles during tumorigenesis. For instance, TLE1 coordinated with Qin to promote cell growth and agar colony formation in chicken embryo fibroblasts [39]. TLE2 was discovered to bind with replication and transcription activator (RTA) and thus inhibited RTA-mediated replication and transactivation that was implicated with Kaposi’s sarcoma-associated herpesvirus [40]. TLE1 and TLE4 served as a tumor suppressor gene in acute myeloid leukemia [41, 42], while it turned to be oncogenes in lung cancer and colorectal cancer, respectively [43–45]. Another member of TLE family, the TLE3 also performs various roles in cancers, especially in clinical treatments containing taxane therapy as mentioned above. On the one hand, TLE3 was found elevated in cervical neoplasms [23, 24], high-grade meningiomas [26], and prostate tumor [27, 28]. On the other hand, high expression of TLE3 was associated favorable responses to taxane-containing therapies in ovarian carcinoma [31] but not in breast cancer [32] and angiosarcoma [46]. Noteworthy, Zagouras P et al. reported that TLE family proteins were up-regulated in colonic adenocarcinoma as detected by panTLE antibody that recognized the entire TLE family [23], whereas our study showed that TLE3 was down-regulated in CRC. In addition, previous studies have showed hyper-methylation of TLE3 [25] and overexpression of TLE4 in CRC [43]. Taken together, we inferred that it was TLE4, TLE1 and TLE2 but not TLE3 that were overexpressed in colonic adenocarcinoma. The multiple properties of TLE family were explained by context-dependent characteristics [17], but the underlying mechanism remains largely unknown and emerge great potential in cancer research.

As an element of Notch signaling that regulates cell fate determination, TLE3 participates in cell differentiation under physiological circumstance [21, 47–51]. As for CRC cancer, we observed that TLE3 could cause the G1-S phase transition arrest in a certain extent and repress the growth and proliferation of CRC. Both p21 and p27 have been identified as mediators of tumor suppression through G1 or G2 arrest, involving binding to CyclinA/cyclin-dependent kinase (CDK) 2, CyclinE/CDK2, and CyclinD/CDK4/6 complexes [35, 36, 52]. Loss of p21 and p27 could enhance tumorigenesis [53]. Further studies have revealed that Ras/MAPK and PI3K/AKT signaling were closely associated with p21 and p27. On the one hand, Ras/MAPK and PI3K/AKT signaling play vital roles in proliferation partly via the regulation of cyclinD1 and CDK inhibitors including p21 and p27 [54–56]. The ubiquitylation-dependent proteasomal degradation of p21 and p27 is mediated by Ras/MAPK and PI3K/AKT signaling [57]. On the other hand, p27Kip1 promoter could be activated by the FOXO family (FOXO4, FOXO3a, and FOXO1), whose activity was modulated by Ras/MAPK and PI3K/AKT pathways [58–60]. Moreover, Gro is a junction of Ras-associated network of multiple signaling cascades, which could attenuate the Gro-dependent repression [17, 61]. Here, we showed that p-ERK, p-GSK and p-AKT were down-regulated by TLE3, indicating the suppressor role of TLE3 in MAPK and PI3K/AKT pathways. Correspondingly, p21 and p27 protein expression were up-regulated by TLE3. In addition, TLE3 enhanced the transcription of p21 and p27, which could be explained by the contribution of FOXO3a.

## Conclusions

Collectively, our study uncovered another novel aspect of TLE3 in the progression of CRC. Lower expression of TLE3 was closely associated with more advanced CRC progression and poorer outcome of patients with CRC, while overexpression of TLE3 suppressed CRC proliferation both in vitro and in vivo. Furthermore, TLE3 could cause G1-S phase transition arrest by increasing the expression of p21 and p27, the underlying mechanism of which was TLE3-mediated inhibition of MAPK and AKT signaling pathways. These findings indicate the potential of TLE3 as a biomarker for CRC prognosis. However, the detailed mechanism of TLE3 in CRC progression needs further investigations.

## Additional files

Additional file 1: Table S1. Primer Sequences used for RT-qPCR (5’ to 3’). (DOCX 13 kb)
Additional file 2: Figure S1. Gene set enrichment analyses of TLE3 based on TCGA COAD RNA Seq dataset. **a** TLE3 expression negatively was correlated with genes related to cell cycle. **b** TLE3 expression was negatively correlated with genes related to G1-S transition. (PNG 116 kb)
Additional file 3: Figure S2. Statistical analyses of flow cytometry indicated that overexpression of TLE3 caused the arrest of G1-S phase transition (a) and increased apoptosis of CRC cells (c), while knockdown of TLE3 promoted the G1-S phase transition (c) and inhibited apoptosis of CRC cells (d). Error bars represent mean ± SD from 3 independent experiments. * *p* < 0.05. (PNG 202 kb)
Additional file 4: Figure S3. Gene set enrichment analysis of TLE3 based on TCGA COAD RNA Seq dataset showed that TLE3 expression was negatively correlated with AKT activity. (PNG 61 kb)
Additional file 5: Figure S4. RT-qPCR analyses of relative mRNA expression of p21Cip1/WAF1 and p27Kip1 in indicated CRC cell lines. Error bars represent mean ± SD from 3 independent experiments. * *p* < 0.05. (PNG 162 kb)

## Abbreviations

CDK: Cyclin-dependent kinase
CRC: Colorectal cancer
Gro: Groucho
GSEA: Gene set enrichment analysis
HLF: Hepatic leukemia factor
IHC: Immunohistochemistry
MAPK: Mitogen-activated protein kinase
MTT: 3-(4, 5-dimethylthiazol-z-yl)-2, 5-diphenyltetrazolium bromide
p21: p21Cip1/WAF1
p27: p27Kip1
Q: Glutamine-rich
RT: Reverse transcription
RTA: Replication and transcription activator
RTK: Receptor tyrosine kinase
RT-qPCR: Real time quantitative polymerase chain reaction
shRNA: Short hairpin RNA
TCGA: The Cancer Genome Atlas
TLE: Transducin-like enhancer of Split
WD: Tryptophan–aspartate
